# Computational and Mathematical Methods in Medicine Prediction of COVID-19 in BRICS Countries: An Integrated Deep Learning Model of CEEMDAN-R-ILSTM-Elman

**DOI:** 10.1155/2022/1566727

**Published:** 2022-04-04

**Authors:** Qi Zhao, Zhongtuan Zheng

**Affiliations:** School of Mathematics Physics and Statistics, Shanghai University of Engineering Science, Shanghai 201620, China

## Abstract

Since the outbreak of COVID-19, BRICS countries have experienced different epidemic spread due to different health conditions, social isolation measures, vaccination rates, and other factors. A descriptive analysis is conducted for the spread of the epidemic in the BRICS countries. Considering the nonlinear and nonstationary characteristics of COVID-19 data, a principle of decomposition-reconstruction(R)-prediction-integration is proposed. Correspondingly, this paper constructs an integrated deep learning prediction model of CEEMDAN-R-ILSTM-Elman. Specifically, the prediction model is integrated by complete ensemble empirical mode decomposition (CEEMDAN), improved long-term and short-term memory network (ILSTM), and Elman neural network. First, the data is decomposed by adopting CEEMDAN. Then, by calculating the permutation entropy and average period, the decomposed eigenmode component IMFs are reconstructed into four sequences of high, medium, low level, and trend term. Thus, ILSTM and Elman algorithms are used for component sequence prediction, whose results are integrated as the final results. The ILSTM is established based on the LSTM model and the improved beetle antennae search algorithm (IBAS). The ILSTM mainly considers that the prediction accuracy of LSTM model is vulnerable to the influence of parameter selection. The IBAS with adaptive step size is used to automatically optimize the super parameters of LSTM model and to improve the modeling efficiency and prediction accuracy. Experimental results indicate that compared with other benchmark models, CEEMDAN-R-ILSTM-Elman integrated model predicts the number of newly confirmed cases of COVID-19 in BRICS countries with higher accuracy and lower error. Strict social policies have a greater impact on the infection rate and mortality rate of the epidemic. During July-August 2021, epidemic spread in BRICS countries will slow down, and the overall situation is still quite severe.

## 1. Introduction

Since the beginning of 2020, the COVID-19 epidemic has swept the world. As of June 22, 2021, the number of confirmed cases of new coronary pneumonia in the world reached 179.43 million, and the cumulative death rate was 3.88 million, with a mortality rate of 2.165%, which has brought substantial amounts of health, economic, environmental, and social challenges. The cumulative number of confirmed cases of new coronary pneumonia in the BRICS countries reached 50.01 million, accounting for 28% of the world, with a case fatality rate of 1.97%. The B16172 mutant strain that newly appeared this year, named, “Delta Mutant” by the WHO, has spread to about 100 countries around the world. The mutant virus spreads exponentially, making the peak of this round of epidemics in various countries faster than the previous wave. The diagnosis rate of India, South Africa, and Brazil, which have higher population densities and a large base of impoverished population, has reached the top 5 in the world. Because of different age structures, hygienic conditions, and vaccination rates, Brazil, Russia, India, China, and South Africa (BRICS) have different infection and death rates. India, Brazil, South Africa, and Russia reported nearly 50,000, 80,000, 10,000, and 15,000 new cases in a single day for consecutive days, indicating that the spread of the new coronavirus is still accelerating. The cumulative number of confirmed cases of the new crown in India has reached more than 30 million, making it the country with the largest number of infections in the BRICS, with an infection rate of 2.18% and a mortality rate of 1.30%. The peak of the second wave of the epidemic in India has passed, and the transmission rate has slowed down. However, due to factors such as social activities in the country and religious gatherings, the future situation of the epidemic in India is still not optimistic. India, Brazil, and Russia rank second, third, and fourth in the world for confirmed cases of new coronary pneumonia, South Africa is the country with the largest number of confirmed cases of new coronary pneumonia in Africa. Affected by this, the economies of the four countries shrank sharply. Brazil, South Africa, and Russia ushered in the third wave of the epidemic. The prediction of the epidemic is helpful for policymakers to formulate epidemic prevention and control measures. At the same time, it is of great significance for promoting the joint response of the BRICS countries to the challenges of the epidemic and promoting cooperation and development.

Many scholars have made efforts to prevent the epidemic and have proposed a large number of epidemic dynamic models, such as the classic differential equation model to predict the spread of epidemics [1, 2]. Babaei et al. [1] used the susceptible exposure infection recovery (SEIR) model to analyze the impact of health protection measures such as isolation, masking, and social distancing on hypothetical populations. At the same time, they used the Brownian motion process to calculate the environmental noise of the data centre. Campillo-Funollet et al. [3] used SEIR-D quantitative epidemiological modeling for healthcare demand, capacity, and the impact of local outbreaks of COVID-19 predicting, and the model exhibits a high accuracy in the prediction. Savi et al. [2] based on the framework of the SEIR model to analyze different scenarios of COVID-19 in Brazil.

In the study of predicting infectious diseases, especially deep learning methods [4–11], other classic models have been conquered in the short-term estimation of epidemics. Devaraj et al. [4] used autoregressive integrated moving average model (ARIMA), long short-term memory (LSTM) [5], and stacked long short-term memory (SLSTM) to predict the cumulative confirmed cases, death cases, and recovery cases of COVID-19 in India and Chennai. Wang et al. [6] used the built-in rolling update mechanism of LSTM and introduced the diffusion index (DI) to make long-term predictions of the epidemic trend in the three countries of Russia, Peru, and Iran. Abbasimehr and Paki [7] combined deep learning models (CNN and LSTM) with Bayesian optimization algorithms to predict COVID-19 time series data. Kafieh et al. [8] applied multilayer perceptrons, random forests, and different versions of LSTM to predict the epidemic in selected countries. Omran et al. [9] applied LSTM and gated recurrent unit (GRU) on time-series data in three countries: Egypt, Saudi Arabia, and Kuwait. Chimmula and Zhang [10] used a long short-term memory network (LSTM) to predict the end date of the Canadian epidemic. Hasan [11] established an EEMD-ANN model to predict the COVID-19 epidemic, resulting from the COVID-19 data being nonlinear and unstable. Guo and He [12] developed an artificial neural network (ANN) for modeling of the confirmed cases and deaths of COVID-19. The best simulating performance with RMSE, R, MAE is realized using the 7 past days' cases as input variables in the training and test dataset.

At the same time, some scholars have also proposed a combined machine learning model and complex network propagation method to study the relationship between COVID-19 and social isolation, medical conditions, socioeconomic, environmental sustainability, and other influencing factors [13–19]. Zhu et al. [13] and Montes-Orozco et al. [14] built a complex COVID-19 network based on the information of each country. The results showed that the global COVID-19 pandemic network has special complex network characteristics. Jithesh [15] used the cellular automata which initially configured to have only susceptible and exposed states. Enlarged and evolved in discrete time steps to different infection states of the COVID-19 pandemic. Li et al. [16] identified critical factors associated with COVID-19 cases, death, and case fatality rates by using the logistic regression model. Anser et al. [17] developed two broad models to evaluate the impact of environmental sustainability ratings, financial development, and carbon damage on the new COVID-19 cases in a cross-sectional panel of 17 countries. Abdel Hafez and Hamdan [18] used three artificial neural network (feed-forward, NARX, and Elman network [19]) methods to evaluate the relationship between weather variables and COVID-19 cases.

Existing research mainly focused on how to apply various algorithm models to COVID-19 prediction, ignoring the optimization of the model. At the same time, it is difficult for shallow machine learning algorithms to fully dig out the underlying essential features of case data and ignore the potential connection between epidemic data and influencing factors, leading to the problem of unsatisfactory prediction results. And the current research pays little attention to the comparative analysis and research of the COVID-19 epidemic in strategic cooperation countries such as the BRICS countries. This article is the first time to study the prediction and analysis of the epidemic situation in the BRICS countries. Compared with the existing COVID-19 prediction models, the integrated CEEMDAN-R-ILSTM-Elman model proposed in this paper has the following advantages.

1. Conduct a descriptive analysis of the spread of the epidemic in the BRICS countries, as well as Spearman's correlation analysis of the influencing factors of the epidemic and analyzed the impact of strict social policies and vaccination on the epidemic
2. Use CEEMDAN to decompose the number of new cases with nonlinear changes and noise characteristics into multiple stable subsequences step by step, which solves the problem of modal aliasing and the improper addition of white noise amplitude in EEMD
3. Calculate the permutation entropy value and average period value of each modal component IMF, and carry out sequence reconstruction, which is divided into four sequences of high, medium, low level, and trend items. According to the reconstructed components, it is possible to better analyze the influence of each influencing factor on the spread of the epidemic and effectively reduce the error caused by multisequence prediction
4. Use ILSTM and Elman algorithms to predict the high-level trend items, and mid- and low-level components, respectively, and use the improved beetle antennae search algorithm to obtain the best hyperparameters (the number of hidden layer units, batch size, and learning rate) automatically for the long short-term memory network model, effectively improving the prediction accuracy and modeling efficiency
5. Integrate and predict the number of newly confirmed cases in India, South Africa, Brazil, Russia, and China through the simple addition (ADD) method, use different evaluation indicators to evaluate the prediction accuracy of the model, compare it with benchmark models such as ARIMA to determine the number of best hidden units and the initial learning rate value of the maximum prediction accuracy. This article uses the adaptive beetle antennae Search algorithm to optimize the number of two hidden layer units, the batch size, and learning rate of each LSTM model according to the update of the step length and the distance between the two whiskers. The Adam algorithm is used to train the model. So that reduce the workload of manual tuning and ensure the accuracy of the forecast. And predict the number of new cases in each country in the next two months

## 2. Materials and Methods

### 2.1. CEEMDAN Algorithm

Empirical mode decomposition (EMD) and ensemble empirical mode decomposition (EEMD) can also be considered as very useful tools for analyzing data with high complexity and irregularity. Huang et al. [20] proposed EMD decomposition, which decomposed noisy data according to its own time-scale characteristics, without presetting any basis functions, and had obvious advantages in processing nonstationary and nonlinear data. The EEMD (Ensemble Empirical Mode Decomposition) algorithm is based on the EMD algorithm by adding normally distributed white noise to the original signal, so that the signal is evenly distributed at the extreme points of the entire level band, which reduces the mode mixing effect [21]. The CEEMDAN algorithm adds limited adaptive white noise based on EEMD, which overcomes the incompleteness and reconstruction error of EEMD after adding white noise [22]. The CEEMDAN-based data processing hybrid model is beneficial to improve the prediction accuracy of the algorithm [23, 24]. The specific implementation steps of this algorithm are as follows.

**Step 1 .**

Add the white noise *v*^*i*^(*t*) obeying the standard normal distribution to the original signal *S*(*t*), and the *i*th signal is expressed as: *S*^*i*^(*t*) = *S*(*t*) + *v*^*i*^(*t*), *i* = 1, 2 ⋯ , *I*. The EMD experimental signal *S*^*i*^(*t*) is decomposed into *IMF*_1_ = 1/*I*∑_*i*=1_^*I*^*IMF*_1_^*i*^. The residual signal is *r*_1_(*t*) = *S*(*t*) − *IMF*_1_.

**Step 2 .**

Add white noise *r*_1_(*t*) to the residual *v*^*i*^(*t*), perform *i* experiments, and use EMD to decompose each experiment into *r*_1_^*i*^(*t*) = *x*(*t*) + *v*^*i*^(*t*). Obtain its first-order component *IMF*_2_ = 1/*I*∑_*i*=1_^*I*^*IMF*_1_^*i*^ and residual signal *r*_2_(*t*) = *S*(*t*) − *IMF*_2_.

**Step 3 .**

Repeat the above decomposition process to obtain the IMF components and the corresponding residuals that meet the conditions. When the residual is a monotonic function and cannot be decomposed by EMD, the program terminates. The final original signal and residual signal can be expressed as *S*(*t*) = ∑_*i*=1_^*n*^*IMF*_*i*_ + *r*_*n*_(*t*) and *r*_*n*_(*t*) = *S*(*t*) − ∑_*i*=1_^*n*^*IMF*_*i*_.

### 2.2. Permutation Entropy Space Reconstruction Algorithm

In this paper, Permutation Entropy (PE) proposed by Bandt and Pompe is used to detect the randomness and dynamic changes of time series [25]. PE has the advantages of simple definition, fast calculation speed, and good robustness. The algorithm is briefly described as follows. Consider the time series {*x*(*i*), *i* = 1, 2, ⋯, *N*}, the length is *N*. It can be reconstructed in phase space as

(1) $$\begin{array}{c} X\left(i\right)=\left\{x\left(i\right),x\left(i+\lambda \right),\cdots x\left(1+\left(m-1\right)\lambda \right)\right\}, \end{array}$$

where *m* is embedding dimension, and *λ* is the time delay. Rearrange each reconstruction component in ascending order as

(2) $$\begin{array}{c} X\left(i\right)=\left\{x\left(i+\left(j_{1}-1\right)\lambda \right)\leq x\left(1+\left(j_{m}-1\right)\lambda \right)\right\}, \end{array}$$

(3) $$\begin{array}{c} i=1,2,\cdots ,N-m+1. \end{array}$$

The column index of each element in the vector constitutes a sequence of symbols:*S*(*g*) = [*j*_1_, *j*_2_, ⋯*j*_*m*_], where *g* = 1, 2, ⋯, *k*, *k* ≤ *m*!, there are a total of *m* types of symbol sequences with different *m*! dimensional phase space mapping. Calculate the number of occurrences of each symbol sequence divided by the total number of occurrences of *m*!different symbol sequences as the probability of the symbol sequence. The probability distribution is *P*(*g*) = [*P*_1_, *P*_2_ ⋯ *P*_*K*_]. The permutation entropy of time series {*x*(*i*)} can be defined as the entropy of *k* different symbols:

(4) $$\begin{array}{c} H_{p}\left(m\right)=-\overset{k}{\underset{g=1}{\sum }}p_{g}\ln p_{g}. \end{array}$$

Note that when *P*_*j*_ = 1/*m*!, *H*_*p*_(*m*) reaches its maximum value. For convenience, *H*_*p*_(*m*) can be normalized to 0 ≤ *H*_*p*_ = *H*_*p*_(*m*)/ln(*m*!) ≤ 1 by ln(*m*!). In fact, *H*_*p*_ can effectively represent the randomness and dynamic changes of the time series. The smaller the *H*_*p*_ value, the more regular the time series. The larger the value of *H*_*p*_, the more random the time series. Some studies reconstruct the IMFs decomposed from sample data into high and low-frequency sequences according to the PE value [26].

### 2.3. LSTM Network Optimized Based on the Improved Long-Term Beetle Algorithm

#### 2.3.1. Beetle Antennae Search

BAS algorithm (beetle antennae search-BAS) is an optimization algorithm based on the principle of bionics and by imitating the foraging behavior of long-term beetle in nature [27]. Compared with other intelligent optimization algorithms such as particle swarm algorithm and bird swarm algorithm. BAS algorithm only needs one beetle individual to perform optimization. Each iteration is faster, which greatly reduces the overall running time of the algorithm without limiting the specific form of the fitness function. The BAS algorithm means that the beetle individual finds the global optimal solution through a continuous trial and update of the individual's position in the solution space. In dimension *D*, the beetle heading vector is represented and normalized as

(5) $$\begin{array}{c} \overset{⟶}{b}=\frac{\mathrm{rand}\left(k,1\right)}{\left\|\mathrm{rand}\left(k,1\right)\right\|}, \end{array}$$

where *m* is the number of iterations, *x*_*rt*_ and *x*_*lt*_, respectively, represent the spatial coordinates of the right and left beetles at the *m*th iteration; *d* represents the distance between the left and right beetle antennae. It can be set according to the step length:

(6) $$\begin{array}{c} \left\{\begin{array}{c} x_{rt}=x^{m}+d\cdot \overset{⟶}{b},\\ x_{lt}=x^{m}-d\cdot \overset{⟶}{b}. \end{array}\right. \end{array}$$

According to the fitness function, the fitness value of the left and right beetle antennae in the current space is judged. *f*(*x*_*rt*_) and *f*(*x*_*lt*_) are the fitness functions. To imitate the detection mechanism of the long beetle, the following position update iterative model is generated:

(7) $$\begin{array}{c} x^{m+1}=x^{m}+\delta^{m}\cdot \overset{⟶}{b}\cdot \mathrm{sign}\left(f\left(x_{rt}\right)-f\left(x_{lt}\right)\right). \end{array}$$

#### 2.3.2. Improved Beetle Algorithm (IBAS)

When the original BAS algorithm with a fixed step is applied, the global search and local search process have relatively general search speed and accuracy problems. To solve this problem, this paper uses a variable step search method based on exponential decay [28]. When it is at the initial position, it is often far from the true solution. Therefore, the initial step size is set to be large and begin to be reduced as the beetle goes forward. Since the step size is proportional to the individual size of the beetle, in the initial stage, the beetle will take big steps to improve the global search ability. In the later period of the iteration, the small beetle will take small steps to improve the local search ability. At the same time, the basic resolution step_0_ is adopted, and the exponential attenuation gradually tends to 0, which is not conducive to the local search under high iteration times. Therefore, the basic step size is set as the basic resolution, and the following update step size is used:

(8) $$\begin{array}{c} \text{step}=e^{-ut}\text{step}+{\text{step}}_{0}. \end{array}$$

The attenuation coefficient *u* and step_0_ are set according to physical truth. The selection of the search step will fall into the local optimum in the iterative process. To make the algorithm jump out of the local optimum, the Monte Carlo criterion of simulated annealing (SA) is used to improve the BAS algorithm [29]. SA simulates the annealing process of the object, which searches the lowest energy and the optimal value of the target. Simulated annealing introduces random factors in the process of searching and optimizing, that is, accepting an inferior solution with an appropriate probability to reduce the probability of falling into the local optimum. The Monte Carlo criterion is used to improve the BAS algorithm. In the iterative process, the inferior solution is accepted with probability *p*, thereby improving the global optimization ability of the BAS algorithm.

(9) $$\begin{array}{c} p=\left\{\begin{array}{c} 1\;f\left(x^{m}\right)<f\left(x^{m-1}\right),\\ \exp\left(-\frac{f\left(x^{m}\right)-f\left(x^{m-1}\right)}{T}\right)f\left(x^{m}\right)<f\left(x^{m-1}\right). \end{array}\right. \end{array}$$

In the formula, *f*(*x*^*m*^) represents the fitness function value at the preupdate position; *f*(*x*^*m*−1^) represents the optimal fitness function value before; exp represents the natural index; *T* is the higher temperature. Because the cooling rate determines the ability to accept inferior solutions, which directly affects the improved BAS algorithm, the ability of to jump out of the local optimal solution to find the global optimal solution. As the number of iterations continues to increase, the cooling rate of the temperature *T* is very fast, and the difference between *f*(*x*^*m*^) and *f*(*x*^*m*−1^) fluctuates less. Therefore, as the iteration progresses, the probability of accepting the inferior solution *p* will gradually decrease.

#### 2.3.3. LSTM Network Model Optimized Based on IBAS Algorithm

When using LSTM model to predict, manual tuning and optimization will greatly reduce the modeling efficiency. How to automatically select the most suitable time window for the subparameter sequences with different level distributions is also an important factor affecting the forecast accuracy. This study uses the improved beetle antennae search algorithm to optimize the long and short-term memory network model for prediction. The ILSTM model construction process is shown in Figure 1.

1. Determine the optimization dimension *K* of the long-term and short-term memory network model according to the long and short-term memory network model
2. Set the hyperparameter value range and iteration termination conditions; use the random function to determine the initial position *x*_0_ of the beetle, and initialize the beetle parameters; set the attenuation index coefficient *u* in the step update formula, the initialization step step, and the basic resolution step_0_, the initial temperature and the individual size ratio coefficient of the beetle, the maximum number of iterations, etc.
3. Set the number of iterations *m* = 0, and set the optimal position *x*_best_ = *x*^0^; set the optimal fitness value with *f*_best_ = *f*(*x*_best_)
4. Calculate the left and right antennae coordinates *x*_*lt*_ and *x*_*rt*_ of the individual long beetle; construct a long and short-term memory network model according to the coordinate values of the left and right antennae, and train the data sets of the prediction problem, and then calculate the fitness value *y*_*lt*_ and *y*_*rt*_ of the right and left antennae of the long beetle according to the objective function; update the beetle step length according to formula (8)
5. According to the acceptance probability *p*, judge whether to update the optimal position of the beetle. If ‖*f*(*x*^*m*^)‖_2_ ≥ ‖*f*_best_‖_2_, to update the optimal position of the beetle when rand < *p*, that is, *x*_best_ = *x*^*m*^, *f*_best_ = *f*(*x*^*m*^); otherwise, do not update, discard bad value of the current beetle position, maintain the last beetle position value *x*^*m*^
6. Repeat formula (2)~(6) until the conditions of iteration number are satisfied. It is considered that the algorithm has generated the optimal solution and updated the optimal solution as *x*_best_; use the hyperparameters corresponding to the optimal solution (the LSTM unit number of each hidden layer, batch size, and learning rate) to build a long and short-term memory network model

### 2.4. New Case Prediction Model Based on CEEMDAN-R-ILSTM-Elman

The basic framework of CEEMDAN-R-ILSTM-Elman prediction model is shown in Figure 2.

1. *Data Decomposition*. Decompose the time series data of new cases into several IMFs series and residual series through CEEMDAN algorithm
2. *Reconstruction Sequence*. Calculate the permutation entropy and average period, and divide it into high-level, medium-level, low-level, and trend series
3. *Component Prediction*. Use the long and short-term memory network model optimized by the IBAS algorithm to predict the high-level components and trend items, and the Elman neural network is used for the medium-level and low-level components
4. *Integrated Prediction*. The final prediction result of the original time series data *x*_*t*_ can be expressed as ${\overset{⌢}{x}}_{t}=f\left({\hat{d}}_{t}\left(1\right),{\hat{d}}_{t}\left(2\right),\cdots {\hat{d}}_{t}\left(K\right)\right)$, where ${\hat{x}}_{t}$ represents the final prediction result at time *t*, ${\hat{d}}_{t}$ is the individual predicted value of the *j*th component, and $f\left({\hat{d}}_{t}\right)$ is the function of ensemble prediction. A simple and effective addition (ADD) strategy is used to aggregate four separate prediction results ${\hat{d}}_{t}\left(j\right)\left(j=1,2\cdots ,k\right)$ to obtain the final combined prediction. The optimal weight of the ADD method is 1 : 1 : 1 : 1

## 3. Results and Discussion

### 3.1. Data Set and Evaluation Indicators

In this paper, the data of newly confirmed cases of COVID-19 in the BRICS countries are obtained from Google Cloud Platform (https://github.com/owid/covid-19-data) collection. The sampling period is from January 23, 2020, to June 22, 2021, and a total of 517 observations. The data accounting for 85% of the observation value are used for model training. The remaining 15% of the samples are used as the test set, and different statistical methods are used to evaluate the effectiveness of each model.

In order to evaluate the loss error of model prediction accuracy, root mean square error (RMSE) and mean absolute percentage error (MAPE) are used. The formulas are as follows:

(10) $$\begin{array}{c} \text{MAPE}=\frac{1}{N}\overset{N}{\underset{t=1}{\sum }}\left|\frac{x_{t}-\overset{\wedge }{x_{t}}}{x_{t}}\right|, \end{array}$$

(11) $$\begin{array}{c} \text{RMSE}=\sqrt{\frac{1}{N}\overset{N}{\underset{t=1}{\sum }}{\left(x_{t}-\overset{\wedge }{x_{t}}\right)}^{2}}, \end{array}$$

where *x*_*t*_ represents the actual value, ${\overset{\wedge }{x}}_{t}$ is the predicted value of the sample data at time *t*, and *N* is the size of the test set. When the error between MAPE and RMSE becomes smaller, it proves that the prediction accuracy of the evaluation model is higher.

In addition to the horizontal prediction accuracy, another key measure of prediction performance is the directional prediction accuracy, which is evaluated by the directional statistics (*D*_stat_) [30].

(12) $$\begin{array}{c} D_{\text{stat}}=\frac{1}{N}\overset{N}{\underset{t=1}{\sum }}a_{t}\times 100\%. \end{array}$$

When $\left({\overset{⌢}{x}}_{t+1}-x_{t}\right)\left(x_{t+1}-x_{t}\right)\geq 0$, *a*_*t*_ = 1, otherwise, it equals to 0.

### 3.2. Descriptive Analysis of the Epidemic

#### 3.2.1. Analysis of the Severity of the Epidemic

India, South Africa, and Brazil have relatively high population densities, a large base of poor population, insufficient medical conditions and capabilities, and cannot meet certain conditions such as isolation, nucleic acid testing, and vaccination. This chapter compares and analyzes the epidemic in the BRICS countries from four aspects: infection rate, mortality rate, reproduction rate, and vaccination rate. The results are shown in Figure 3.

From the big outbreak in March 2020 to June 22, 2021, among the BRICS countries, the total number of cases per million people, the total number of deaths per million people, and the infection rate reached the highest in Brazil, at 84939.326 and 2374.475. It shows that Brazil's epidemic situation is the most severe. Russia and China have relatively advanced medical and health standards and relatively low mortality rates. The number of people vaccinated per 100 people in China reached the highest at 74.46, and South Africa reached the lowest at 3.97. The total number of vaccinated people was less than 2.5 million, and the reproduction rate reached the highest at 1.37. It is the most severely affected country on the African continent. The vaccination rate in India is 21%. Because India and South Africa have large populations and poor medical and health conditions, they cannot reach a certain vaccine level in a short time. Due to the invasion of the Delta variant, the number of confirmed cases and deaths currently experienced by India, South Africa, and Brazil is still rising at an unprecedented rate.

#### 3.2.2. Spearman Correlation Test of Factors Affecting the Epidemic

To better analyze and predict the epidemic trend of COVID-19, this section uses Spearman correlation analysis to capture the COVID-19 infection rate and mortality rate and influencing factors (average age of the population, handwashing facilities, number of beds per 1,000 people, and vaccination rate et al.). The Spearman correlation is used to capture the correlation between variables, which ranges from -1 to +1. The Spearman correlation coefficient is calculated as the product of the covariance of the two variables divided by the standard deviation of each data sample, which normalizes the covariance between the two variables to give an interpretable score. The Spearman correlation test results are shown in Figure 4.

The analysis of the correlation heat map shows that the COVID-19 infection rate depends on the two characteristics of handwashing facilities and strict social measures, and the correlation coefficients are -0.65 and -0.67, respectively. The more handwashing facilities, the lower the infection rate, because there are a large number of slum areas in India, South Africa, and Brazil, and sanitary facilities such as handwashing are extremely backward. Strict social measures have reduced large-scale gatherings and reduced the infection rate. Mortality is strongly correlated with GDP per capita, extreme poverty index, handwashing facilities, beds per 1,000 people, and vaccination rates. The correlation coefficients are -0.52, -0.85, -0.65, and -0.67. It shows that medical conditions have a very high impact on the mortality rate. If the economy is low, it is impossible to purchase a large number of vaccines, resulting in a low vaccination rate and resulting in the death rate cannot be reduced. Handwashing facilities are one of the most important measures, which have a greater impact on reducing infection rates and mortality. However, the relationship between vaccination rate and infection rate is weak, because the current vaccination rate is low and the impact on the infection rate is relatively low.

#### 3.2.3. Analysis of the Impact of Strict Social Policies on the Epidemic

In many cases, people infected with COVID-19 do not have any symptoms in the early stages, so they do not know their condition and continue to interact with other people. Travel restrictions and facility closures can prevent them from contacting others and spreading the coronavirus to a certain extent, but they cannot completely prevent them. Social distancing measures require everyone to stay indoors. Therefore, social distancing measures are considered the most effective measures to prevent infection in the community. This article analyzes the impact of strict social policies and vaccination in the BRICS countries on the spread of the epidemic. The result is shown in Figure 5.

According to the above analysis results, after the implementation of strict social measures, the number of COVID-19 cases confirmed daily has decreased. Within one month after the implementation of the most stringent socially strict measures, the number of daily confirmed cases in most countries reached a peak and began to decline. It can be observed that the number of months from the first two rounds of outbreaks to recovery in South Africa, Brazil, India, and Russia was 4, 4, 5, 1, and 2, 3, 2, and 2, respectively. At the same time, the time required for daily deaths to decline is 2 weeks slower than the time required for daily confirmed cases in these countries to start to decline. The effectiveness of strict social measures on the spread of COVID-19 differs among the 5 countries. This difference may be due to the different levels of time intervals of the strict social measures promulgated.

In South Africa, with the implementation of level one to three levels of social measures, the number of new cases per day decreased rapidly after reaching the peak. At the same time, the interval between the peaks of the three outbreaks in South Africa is 6 months, and the peak of the second round of new cases is 1.58 times that of the first round. In India, due to the mutation of the virus, rapid transmission, and strong infectivity, the daily highest case of the second round of the epidemic was 4.23 times that of the first round, and the number of deaths also reached 3.68 times, resulting in the effect of social distancing measures on the interruption of the epidemic is weak. In Brazil, due to the government's failure to issue social distancing measures in a timely manner and the implementation of social distancing measures at a low level, this resulted in a large-scale outbreak of the epidemic, which was severe throughout the year. The peak of new cases in the third round was 1.43 times that of the first round. The peak of death cases was 2.48 times that of the first round. This may be due to the mutation of the virus.

With the start of vaccination work in various countries, the population of the first phase of vaccination will be antimedical personnel and front-line workers. Russia started vaccination in December last year at the earliest, so the Russian epidemic situation has slowed down since then. India's low vaccination rate due to the popular Big Kettle Festival and other reasons led to the second major outbreak of the epidemic. Brazil and South Africa's new coronavirus vaccination programs are being promoted among middle-aged and elderly people, and the average age of patients who die from the new coronavirus has dropped.

### 3.3. CEEMDAN Decomposition and Reconstruction of New Case Data

To overcome the problems of EMD and EEMD modal aliasing, the CEEMDAN algorithm adds adaptive Gaussian white noise at each stage of the new case data, and the original new case can be decomposed into multiple modal components by calculating. The decomposition process is complete, and the error is extremely low. We use the MATLAB tool to decompose the data of new COVID-19 cases in various countries by CEEMDAN, select the appropriate noise standard deviation, the number of implementations, and the maximum number of screening iterations allowed, so that the CEEMDAN decomposition results of the new cases in BRICS countries are obtained as shown in Figure 6.

After decomposing the original data of COVID-19 by CEEMDAN, the unstable and nonlinear characteristics of the data have been arranged in order from the highest level to the lowest level. The original sequence is decomposed into 7or 8 subsequences and a trend component, which are independent of each other. IMF1-3 seems to just randomly walk around zero, which is a high-level component of the series of new daily cases. Except for the trend item, the other IMFs exhibit a certain cyclical nature which are different from each other.

The reconstructed component sequence can reveal the main characteristics of the daily data fluctuation of new COVID-19 cases, determine the movement law of the reconstructed sequence, the influencing factors, and give an explanation. First, calculate the total number of maximum points and minimum points for each IMF within the range of the sample space, and then divide the total number of points in the sample space (days) by the total number of maximum points and minimum points as the average period. Because the residual sequence is a monotonous overall trend, there is no periodicity. For the complexity feature, the PE measurement is used to calculate the permutation entropy value, in which the embedding dimension and time delay are set to 4 and 1. The complexity and periodicity analyses of IMFs of new cases in BRIC countries are shown in Tables 1–5.

It can be seen from Tables 1–5 that the PE value of each country's sequence decomposed by CEEMDAN from IMF1 to the residual gradually decreases from about 1.0 to 0.1. For the data decomposed in South Africa, the PE values of IMF1-4 are all above the threshold value of 0.8, indicating that these sequences may have a higher degree of complexity. The PE value of IMF5 is a threshold between 0.5-0.7, indicating that the sequence may have relatively medium complexity. In contrast, IMF6-9 and residuals are at a relatively low level of complexity because their PE values are below the threshold 0.5. Similar results can be found for the Indian data, that is, the IMF1-4 test is highly complex because the PE value is higher than 0.7, while the IMF5-6 is between 0.5 and 0.7, and the IMF7-8 and the residual are relatively regular. The same is true for Brazil, India, China, and Russia. For the signal period characteristics, the average period of the high-level sequence IMF1-4 is about 15 days for the data of South Africa and India, the average period of the medium level sequence IMF5 is less than 2 months, and the low-level sequence IMF6-9 is greater than 60 days. Each IMF is reconstructed into four types of sequences with different complexity and periodicity to avoid directly using IMFs sequence prediction, error amplification, and cyclic mixing. The reconstructed sequence of each level component is compared with the initial sequence, and the fluctuation characteristics of the reconstructed sequence are also compared. The results are shown in Figure 7.

As shown in Figure 7, the trend item is the most important component in analyzing the long-term trend of new COVID-19 case data, and it plays a decisive role in long-term fluctuations. The upward trend component is synchronized with the trend growth of the new case data. Although the new cases will fluctuate greatly due to the influence of social isolation and medical level, the trend item represents the long-term trend of new cases that is not affected by other factors.

For low-level components, the period is approximately 7.2 months. It can be seen from the figure that the trend of the low-level sequence is consistent with the newly added case sequence. And each fluctuation point corresponds to the peak of new cases in each round of the epidemic. Separating low-level sequences is essential for predicting the number of new cases. The reconstructed low-level sequence can effectively reflect the long-term fluctuations in the data of the new COVID-19 cases. This paper believes that the low-level sequence mainly reflects fixed factors such as medical level, population density, and handwashing facilities.

For medium-level components, the period is about 1-2 months. It can be seen from the graph that the IF sequence is shaped as a sine or cosine wave, matching the different levels of social distancing measures in place at each stage. This paper argues that the intermediate frequency series mainly reflects social isolation measures and variable factors such as accidental importation and large-scale religious gatherings or marches.

For high-level components, the period is about half a month. Although the high-frequency component has little effect on the new cases of COVID-19, with high volatility and insignificant regularity, its cumulative effect cannot be ignored. With the mutation of the COVID-19 virus and the universal vaccination of vaccines, due to the current implementation of phased vaccination policies in various countries, medical staff and the elderly are generally given priority for vaccination to reduce the transmission rate and case fatality rate, and the cumulative impact of short-term fluctuations is increasing.

### 3.4. Analysis of Prediction Results and Model Selection of Each Sequence

#### 3.4.1. Model Parameter Settings

This article selects about 85% of the new COVID-19 cases in each of the BRICS countries for model training, and the rest is used for testing about 15% of the total data. Using the adaptive beetle antennae search algorithm to optimize the number of two hidden layer units, the batch size and learning rate of each LSTM model of the high, medium, low level, and trend items, so that reduce the workload of manual tuning and ensure the accuracy of the forecast. The Adam algorithm is used to train the model. The value range of hyperparameters is set as follows: the number of hidden layer units value range [10,50], the batch size value range [1,64], and the learning rate value range [0.0001,0.002]. The optimization dimension of the adaptive beetle antennae search algorithm is 4, and the initial step size is 1. Set the maximum number of iterations of the beetle antennae search algorithm to 100. The mean absolute error function of the training set is used as the fitness function. Elman algorithm uses trainingdx function for training.

#### 3.4.2. Performance Analysis of the Improved Beetle Antennae Search Algorithm

To further compare the advantages and disadvantages of the BAS algorithm and the IBAS algorithm, this paper selects the high-level sequence to test the model.  Figure 8 shows the optimal iterative convergence curves of the two algorithms. At the same time, the accuracy of the model is described from the three perspectives of root mean square error (RMSE), mean absolute percentage error (MAPE), and the CPU running time during the iteration. The results are shown in Table 6.

It can be seen from Figure 8 that the IBAS algorithm achieves ideal accuracy at approximately 42nd iteration, and the BAS algorithm also achieves the optimal solution at the 55th iteration. The single iteration time of IBAS algorithm is much shorter than that of BAS algorithm, which shows that IBAS converges faster. From Table 6, it can be concluded that the overall running time of the IBAS-LSTM (ILSTM) algorithm and BAS-LSTM is about 200.5 s and 180.6 s. From the perspective of model prediction accuracy, the fitting results of the IBAS-LSTM algorithm are better than the other two algorithms. The percentage error MAPE is reduced by about 1.7% and 3.7%. Therefore, the use of the improved BAS algorithm to optimize the LSTM network effectively solves the problems of the traditional LSTM algorithm, such as the large random initial value, easy to fall into the local optimum, and slower convergence. According to the optimization process in Section 2.3.3, the hyperparameters of each submodel are optimized, and the results are shown in Table 7. At the same time, the relevant parameters of Elman are shown in Table 8.

#### 3.4.3. Comparative Analysis of Each Sequence Prediction Model

To verify the superiority of the combined prediction model compared to other models, the high, middle, low level, and trend components are trained and verified using different benchmark models, Elman, ARIMA, LSTM, ILSTM, and the results are as follows shown in Figure 9.

As shown in Figure 9, by using Elman, ARIMA, LSTM, and ILSTM to train and verify the high, middle, low level, and trend components of new cases in various countries, it can be concluded that the model fitting effect is the best when the ILSTM model is used to predict the high level and trend components, and the Elman model predicts the medium and low-level components.

### 3.5. Analysis of the Prediction Results of the Integrated Model

This paper adopts the root mean square error (RMSE), mean absolute percentage error (MAPE), and direction statistics (*D*_stat_), respectively, to compare the prediction accuracy of proposed CEEMDAN-R-ILSTM-Elman model with CEEMDAN-R-LSTM-Elman, CEEMDAN-R-LSTM-ARIMA, CEEMDAN-R-ILSTM, CEEMDAN-R-LSTM, and CEEMDAN-R-Elman for new COVID-19 cases in various countries. The evaluation index results of each model are shown in Tables 9–11.

In South Africa, compared with the CEEMDAN-R-LSTM-Elman, the RMSE and MAPE of CEEMDAN-R-ILSTM-Elman prediction model have been reduced by 20.73% and 21.64%, respectively, and the directional accuracy indicators have increased by 8.24%. The RMSE and MAPE of CEEMDAN-R-ILSTM, compared with the CEEMDAN-R-LSTM model, are reduced by 6.94% and 5.12%, respectively, and the directional accuracy is increased by 4.7%. It indicates that the optimization speed and prediction accuracy of high-level sequence and trend sequence are effectively improved by optimizing the LSTM model through the IBAS algorithm. Compared with the CEEMDAN-R-LSTM-ARIMA, the RMSE and MAPE values of the CEEMDAN-R-LSTM-Elman model are reduced by 9.75% and 21.87%, respectively, and the directional accuracy index is increased by 3.95%. The Elman decomposition method can effectively improve the prediction accuracy of high, medium, and low-level series, since the traditional linear approach is not suitable for complex nonlinear time-series predictions.

It shows that the CEEMDAN-R-ILSTM-Elman prediction model proposed in this paper improves the efficiency and accuracy of prediction of new COVID-19 cases. Since the fluctuation characteristics of China's epidemic data are greatly affected by various measures, the effect of its model is relatively poor. Finally, the prediction results of the above subsequences are integrated. At the same time, to further confirm the effectiveness of the model in predicting the data of new daily cases with nonlinear and noisy characteristics, the CEEMDAN-R-ILSTM-Elman model proposed in this paper is used for predicting the new cases of COVID-19 in various countries in the next two months, and the results are shown in Figure 10.

As shown in Figure 10, with various social distancing orders and vaccination measures in different countries, the spread of COVID-19 varies greatly among the five countries. The number of new cases in India reached the peak of the second round of the epidemic in May this year, at 418,800, which is 4.23 times the peak of the first wave and will slow down in July or August. The Russian epidemic will usher in the third wave of epidemic peaks in the next between July and August, and daily new cases will increase exponentially. When the peak is equal to the peak of the second wave of about 29,000, it will slow down. At the same time, South Africa will also usher in the third wave of epidemic peaks in the next two months, and the peak will exceed the previous peak of the second wave of epidemics, reaching 1.24 times. The increasing number of new cases in Brazil will start to slow after July. Due to the difficult implementation of Brazil's epidemic policy, the pandemic situation in Brazil will be severe throughout the whole year. The number of new cases reached a peak of 129,025 at the end of June. The failure of countries to implement the universal vaccination policy and social distancing measures in a timely manner caused another major outbreak of the epidemic. In addition to the lower vaccination rate, the delta mutant strain has become an important risk. This strain is more contagious, resulting in a rebound in the epidemic in many countries whose rates of infection and deaths reach its peak again.

Due to economic development, population density, and other social factors, the governments of South Africa, India, and Brazil have been unable to consistently implement the highest-level social distancing measures, support relevant medical facilities, and purchase large amounts of vaccines, it results in the more severe epidemic situation in a global pandemic. In contrast, China began to issue the highest level of social distancing order in one week when the viruses were found and effectively controlled the spread of the virus within three months. Later, due to overseas imports and other reasons, the epidemic rebounded in very few areas, but the spread of the epidemic was quickly contained.

## 4. Conclusions

In view of the nonlinearity and large volatility of the data of the new COVID-19 cases, we propose the CEEMDAN-R-ILSTM-Elman model, which reduces the impact of the original nonstationary sequence on the prediction accuracy and improves the convergence speed and prediction accuracy by comparing with the CEEMDAN-R-LSTM-Elman, CEEMDAN-R-LSTM-ARIMA, and other models. According to the reconstruction components of high, medium, low level, and trend items, it is much better to analyze the influence of social isolation measures, medical conditions, vaccination, and other factors on the spread of the epidemic and effectively reduce the errors caused by multisequence forecasts. The improved beetle antennae search algorithm is used to automatically optimize the hyperparameters of the LSTM model, which effectively improves the prediction accuracy and modeling efficiency.

At the same time, the epidemic situation of various countries in the next two months is analyzed and predicted, although the spread of the epidemic in various countries will slow down in the next two months, the overall situation is still quite severe. In the BRICS countries, the daily new COVID-19 and death cases are affected by the social economy, demographic status, sanitary conditions, strict social policies, vaccination, and other resources and policies. As the virus continues to mutate, countries should strengthen cooperation to reduce socioeconomic inequality and strengthen the operation of the medical and health system to jointly defeat the epidemic. The research will help the five countries to formulate relevant policies to reduce the spread of the epidemic under the current severe situation of the COVID-19 epidemic. In the future, we will conduct dynamic model simulink simulations based on different COVID-19 influencing factors to forecast the spread of the epidemic and contribute to the effective containment of the spread of COVID-19 in the BRICS countries.

## Figures and Tables

**Figure 1:** The structure diagram of the long short-term memory network model optimized by the improved beetle algorithm.

**Figure 2:** The basic framework of the CEEMDAN-R-ILSTM-Elman prediction model.

**Figure 3:** Analysis of infection rate, death rate, reproduction rate, and vaccination rate in each country.

**Figure 4:** Spearman correlation analysis between the factors affecting the epidemic and the infection rate and mortality rate.

**Figure 5:** Analysis of the impact of strict social policies and vaccination rates on new cases and new deaths.

**Figure 6:** CEEMDAN decomposition results of new daily cases. (a) Brazil. (b) Russia. (c) China. (d) South Africa. (e) India.

**Figure 7:** Representation of IMFs reconstruction sequence. (a) South Africa. (b) Brazil. (c) India. (d) Russia. (e) China.

**Figure 8:** Comparison of fitness curves of network models of various optimization algorithms.

**Figure 9:** Representation of the prediction results of each component. (a, c, e, g) South Africa. (b, d, f, h) Brazil. (i, k, m, o) India. (j, l, n, p) Russia. (q, r, s, t) China.

**Figure 10:** Forecast results of the number of new cases in the BRICS countries in the next two months. (a) South Africa. (b) Brazil. (c) India. (d) Russia. (e) China.

**Table 1:** Complexity and periodic analysis of IMFs in South Africa.

Mode	PE value	Complexity	Main timescale
IMF1	0.9943	High level	3.209
IMF2	0.9227	High level	4.872
IMF3	0.8750	High level	5.901
IMF4	0.8081	High level	7.661
IMF5	0.6193	Medium level	18.635
IMF6	0.4656	Low level	73.512
IMF7	0.4326	Low level	118.750
IMF8	0.4123	Low level	197.917
IMF9	0.4014	Low level	475
Residue	0.1032	Trend level	>sample size

**Table 2:** Complexity and periodic analysis of IMFs in Brazil.

Mode	PE value	Complexity	Main timescale
IMF1	0.9907	High level	3.09803
IMF2	0.8835	High level	5.71084
IMF3	0.8588	High level	6.285
IMF4	0.6843	Medium level	20.8979
IMF5	0.6005	Medium level	35.6086
IMF6	0.4141	Low level	112.2954
IMF7	0.4281	Low level	167.416
Residue	0.0611	Trend level	>sample size

**Table 3:** Complexity and periodic analysis of IMFs in India.

Mode	PE value	Complexity	Main timescale
IMF1	0.9978	High level	3.0267
IMF2	0.9704	High level	3.9689
IMF3	0.9543	High level	4.3589
IMF4	0.8608	High level	6.4153
IMF5	0.6832	Medium level	13.975
IMF6	0.5377	Medium level	31.875
IMF7	0.4612	Low level	78.928
IMF8	0.4191	Low level	212.5
Residue	0.1507	Trend level	>sample size

**Table 4:** Complexity and periodic analysis of IMFs in Russia.

Mode	PE value	Complexity	Main timescale
IMF1	0.9934	High level	2.76630
IMF2	0.8413	High level	6.69736
IMF3	0.7113	High level	11.5681
IMF4	0.5635	Medium level	26.7894
IMF5	0.4579	Medium level	78.7738
IMF6	0.4213	Low level	212.083
IMF7	0.3470	Low level	254.065
Residue	0.0211	Trend level	>sample size

**Table 5:** Complexity and periodic analysis of IMFs in China.

Mode	PE value	Complexity	Main timescale
IMF1	0.998	High level	2.85631
IMF2	0.9681	High level	3.9769
IMF3	0.9892	High level	3.4697
IMF4	0.8675	High level	6.0823
IMF5	0.6574	Medium level	14.7714
IMF6	0.5669	Medium level	25.85
IMF7	0.4599	Low level	80.0119
IMF8	0.437	Low level	116.325
IMF9	0.4063	Low level	387.75
Residue	0.096	Trend level	>sample size

**Table 6:** Comparison of different model effects.

Model	RMSE	MAPE	CPU time/s
LSTM	29.26	0.095	125.9
BAS-LSTM	20.38	0.075	180.6
IBAS-LSTM	12.65	0.058	200.5

**Table 7:** Hyperparameters of each sequence model optimized by IBAS-LSTM.

Component	Hidden size *N*1	Hidden size *N*2	Batch size	LearnRate
High level	43.5	24.5	38	0.00165
Medium level	41	28	14.5	0.00075
Low level	31	29.5	53.5	0.0002
Trend level	18	30	47	0.0005

**Table 8:** Hyperparameters of each sequence model optimized by Elman.

Component	Hidden sizes	TrainParam.Epochs
High level	10	100
Medium level	5	100
Low level	5	100
Trend level	8	100

**Table 9:** The prediction error RMSE of each model.

Model	South Africa	India	Brazil	Russia	China
CEEMDAN-R-ILSTM-Elman	8.26	8.89	8.59	7.98	10.56
CEEMDAN-R-Elman	13.39	13.23	13.35	13.47	14.77
CEEMDAN-R-ILSTM	11.96	11.26	12.46	11.21	12.96
CEEMDAN-R-LSTM	12.57	14.15	12.90	12.76	14.23
CEEMDAN-R-LSTM-ARIMA	12.25	13.25	12.18	11.86	13.60
CEEMDAN-R-LSTM-Elman	10.05	10.59	11.09	10.12	12.50

**Table 10:** The prediction error MAPE of each model.

Model	South Africa	India	Brazil	Russia	China
CEEMDAN-R-ILSTM-Elman	0.057	0.059	0.053	0.051	0.078
CEEMDAN-R-Elman	0.082	0.079	0.092	0.090	0.099
CEEMDAN-R-ILSTM	0.072	0.069	0.086	0.084	0.091
CEEMDAN-R-LSTM	0.077	0.073	0.088	0.089	0.095
CEEMDAN-R-LSTM-ARIMA	0.075	0.066	0.079	0.085	0.096
CEEMDAN-R-LSTM-Elman	0.069	0.061	0.062	0.072	0.087

**Table 11:** The prediction accuracy *D*_stat_ of each model.

Model	South Africa	India	Brazil	Russia	China
CEEMDAN-R-ILSTM-Elman	0.82	0.80	0.85	0.79	0.70
CEEMDAN-R-Elman	0.68	0.63	0.64	0.65	0.52
CEEMDAN-R-ILSTM	0.74	0.71	0.71	0.70	0.61
CEEMDAN-R-LSTM	0.71	0.63	0.67	0.61	0.55
CEEMDAN-R-LSTM-ARIMA	0.73	0.62	0.68	0.67	0.58
CEEMDAN-R-LSTM-Elman	0.76	0.72	0.75	0.70	0.64

## Data Availability

The data of newly confirmed cases of COVID-19 in the BRICS countries are obtained from Google Cloud Platform (https://github.com/owid/covid-19-data) collection.
